# Tripartite Evolutionary Game of Agricultural Service Scale Management and Small Farmers' Interests under Government Preferential Policies

**DOI:** 10.1155/2022/4902485

**Published:** 2022-10-10

**Authors:** Kaomin Gou, Luyun Wang

**Affiliations:** ^1^School of Economics, Chongqing University of Finance and Economics, Chongqing 401320, China; ^2^College of Economics and Management, Southwest University, Chongqing, 400715, China

## Abstract

In agricultural production with small farmers as the main body, the service scale operation is one of the ways to obtain scale operation benefits. This paper constructs a tripartite evolutionary game model of agricultural scale service providers (integrators), demand subjects (farmers), and agriculture-related government departments and analyzes the influencing factors, influencing relations, and evolutionary stable equilibrium results of each participant's strategy choice. The results show that improving rewards and punishments and strengthening supervision by agriculture-related government departments will help integrators provide high-quality services and encourage farmers to actively produce and reduce speculation; when the cost difference between high-quality service and low-quality service is large, the probability of high-quality service provided by integrators will be reduced, and the evolution result of low Pareto efficiency may appear in the system; when the speculative cost of farmers is not high, the lobbying efforts of integrators will increase the speculative behavior of farmers. Finally, MATLAB2018a is used to simulate and analyze the validity of the model results, which provides a theoretical reference for the scale operation of agricultural services.

## 1. Questions Raised

Document No.1 of the Central Committee of the Communist Party of China puts forward “developing moderate-scale operation” for 10 consecutive years from 2012 to 2021. The report of the 19th National Congress of the Chinese government also clearly puts forward “developing various forms of moderate-scale operation” in the rural revitalization strategy. Developing moderate-scale operation seems to be the consensus of China's agricultural development. In agricultural production practice and academic research, two agricultural scale operation modes have been explored: land scale operation and service scale operation. Based on the basic national conditions of China with a small population and a large number of small farmers, a large number of scholars believe that Chinese agriculture is more suitable for service scale operation [1–9], that is, small farmers are organized with agricultural socialized services to form a division of labor and cooperation in the agricultural production chain. Small farmers are mainly responsible for agricultural production links, and large-scale service suppliers are responsible for preproduction, mid-production, and postproduction service links; small farmers can share the external “service economies of scale” through the vertical division of labor and service outsourcing of agricultural socialized services, thus realizing the organic connection between small farmers and modern agricultural development [1].

China's agricultural service scale operation practice has been explored for a long time, such as cross-regional service of agricultural machinery [10], and the proprietary concepts of agricultural “service scale operation” and “service scale” were first put forward in the exploration of “land trusteeship” of Shandong supply and marketing cooperatives, and were widely mentioned in the practice of land trusteeship in various places later. With the deepening of academic understanding of the agricultural service scale operation, agricultural service scale operation not only refers to land trusteeship mode but also includes a wider form of agricultural service scale. Mingfeng and Lin [7] believe that the large-scale operation of agricultural services means that there is no transfer of management rights, contracted farmers still maintain the dominant position of independent operation and independent accounting, but through the centralized contiguous land, all or part of the operation links of agricultural production is entrusted to socialized service organizations, and socialized service organizations partially or completely realize agricultural scale operation through the large-scale operation of agricultural production links. This definition highlights “centralized contiguous land,” and the understanding of service scale operation has not yet broken away from the initial exploration trace of land trusteeship. Peng [5] believes that an agricultural service scale operation is a form of agricultural scale operation in which farmers outsource intermediate input services in all aspects of agricultural production and operation, and specialized service providers receive packages and carry out large-scale services. It can be seen that farmers outsource services in production and operation to professional service providers. The relationship between supply and demand that forms the service scale belongs to the scope of service scale operation. It includes the service scale operation generated by land trusteeship and centralized contiguous, the service scale operation formed by the mode of “leading enterprises + professional cooperatives + farmers” in agricultural industrialization, and the service scale operation formed by professional service organizations “professional cooperatives + farmers” or “professional service companies + farmers.”

Scholars have made some research on the service scale operation. Liu [11] pointed out in the question “how to take the road of China's agricultural modernization” that the scale of agricultural services promotes agricultural modernization and realizes the scale of services in all aspects of agricultural production, which can not only improve the profitability of service subjects, but also enable agricultural operators to reduce production costs and form a win-win situation between production subjects and service subjects. Kong and Zhong [12] pointed out that the scale of agricultural services is a beneficial practice of organically combining government forces with market forces to promote the development of modern agriculture by promoting the supply and marketing cooperative system in Shandong Province in “land trusteeship.” Luo [1] pointed out that the essence of service scale operation lies in the division of labor and specialization of agriculture. Once farmers are involved in the socialized division of labor and productive service outsourcing; they can also generate service economies of scale. Zhang [8] studied the service radius of the main body of service scale operation through a case, and pointed out that the decision of service radius is influenced by resource allocation efficiency, geographical environment, market capacity, and main body type. The service scale operation and land scale operation are two interrelated and mutually promoting scale operation strategies [13–15].

However, there are many problems in the scale operation of agricultural services in China. Agricultural professional cooperatives are the main force of socialized services [16] and the main business entities of scale services. However, in practice, there are a large number of “empty shell cooperatives [17–19]” and “pseudo-cooperatives,” and farmers' members have no decision-making power of cooperatives [20, 21], in order to obtain national preferential policies, fiscal expenditure, and tax incentives [22], combined with local government investment promotion policies, and became a profit-making tool for rural minority elites to package speculative capital [20], instead of really serving farmers. There is “elite capture” in the implementation effect of benefiting farmers' policy [18, 23]. “Large farmers dominate, and small farmers are marginalized” [24], the interests of smallholder farmers are not protected [25], and there is an unequal trading relationship between small farmers and large commercial capital [26]; the performance rate of the “contract” between the company and small farmers generally only reaches 20% per month [27]. In the process of farmers' organization and cooperative development, cooperation and confrontation between farmers and organizations always exist [28], and even “cooperation” has become a matter for the government and rural elites, and ordinary farmers are indifferent [29].

In response to the above problems, scholars also put forward a large number of solutions, some proposed to improve the assessment mechanism of cooperatives and the withdrawal of cooperatives according to law [19], and some scholars [24] emphasized the personal ability and altruism of the chairman of cooperatives and their role in “rational cooperatives.” Some scholars have studied the organization of farmers [29] and the interest link mechanism between farmers and service subjects [30]. However, most of the above studies study problems locally and put forward solutions. Few scholars regard the subjects involved in agricultural service scale management as a system, and study the interaction, mutual influence, and evolution results of their behaviors as a whole. Therefore, based on the bounded rationality of each subject of agricultural socialization service, this paper tries to use the tripartite evolutionary game model to discuss it from the perspective of the system as a whole.

## 2. Modeling

### 2.1. The Main Body Involved in the Scale Operation of Agricultural Services and Its Relationship

The scale operation of agricultural services involves subjects, including suppliers, demanders, and regulators of scale services. Scale service providers are the main body of integrated supply of agricultural socialized services from horizontal and vertical dimensions, such as cooperatives, leading enterprises, professional service associations, and professional service companies [5], which are called **integrators** in this paper. In scale service demanders, that is, agricultural producers, including farmers and other new business entities, this paper focuses on the relationship between integrators and farmers, in which scale service demanders are farmers. Finally, it is the supervisor of standardized operation of scale services, including agriculture-related government departments at all levels, such as agricultural committees at city and county levels, poverty alleviation offices, municipal development and reform commissions, municipal supply and marketing cooperatives, rural economic offices at township levels, rural economic management service centers, and agricultural technology service extension service centers. The scale operation of agricultural services involves three subjects and their relationships as shown in Figure 1.

### 2.2. Model Assumptions

In order to study the dynamic evolution of the relationship between the subjects involved in the scale operation of agricultural services, the strategies of all parties, and the evolution equilibrium, this paper makes the following assumptions:

**Hypothesis 1 .**

The three participants, integrators, farmers, and agriculture-related government departments are recorded as participant 1, participant 2, and participant 3, respectively. It is assumed that the participants of the three parties are all bounded rationality, that is, according to the existing practice, they make decisions according to the current situation. The strategy choice gradually evolves and stabilizes in equilibrium strategy with the development of time.

**Hypothesis 2 .**

The policy space of integrators is *α*=(*α*_1_, *α*_2_)= (providing high-quality service and poor-quality service), and choose to provide a high-quality service with the probability of *x* and poor-quality service with the probability of (1 − *x*), *x* ∈ [0,1]. The strategy space of farmers is *β*=(*β*_1_, *β*_2_)=(not speculating and speculating), choosing to join the integrated service organization not speculating with the probability of *y*, choosing to speculate with the probability of (1 − *y*), *y* ∈ [0,1]. The strategy space of government agriculture-related departments is *γ*=(*γ*_1_,*γ*_2_)= (strict supervision and loose supervision), strict supervision is chosen by *z* probability, and loose supervision is chosen by (1 − *z*) probability, *z* ∈ [0,1].

**Hypothesis 3 .**

The integrator gains *R*_1_ from completing the service. If the integrator provides high-quality service, its service cost is *C*_1*h*_, whereas the cost of providing inferior-quality service is *C*_1*l*_ and *C*_1*h*_ > *C*_1*l*_. When integrators provide quality services, there is no need to lobby farmers; when integrators provide inferior services, they need to lobby farmers, and they need to lobby farmers to join the integration organization with immediate small favors and coordinate with each other, which is recorded as lobbying cost *C*_1*c*_. Integrators provide inferior services to generate lobbying costs and speculative costs, such as false propaganda, false information, false staffing, and venue rental. The speculative costs are recorded as *C*_1*s*_ and (*C*_1*c*_+*C*_1*s*_+*C*_1*l*_) < *C*_1*h*_.

**Hypothesis 4 .**

When farmers join the integrated organization, the basic operating income is recorded as *R*_2_. When integrators provide quality services, the income growth of farmers is recorded as *R*_2*i*_. When integrators provide inferior services, the decrease in farmers' income is recorded as *R*_2 *d*_. If farmers join the integrated organization, they will not speculate and generate speculative costs in the business process; otherwise, they will generate speculative costs, which will be recorded as *C*_2_.

**Hypothesis 5 .**

When the government agriculture-related departments formulate strict reward and punishment policies for strict supervision, if integrators provide high-quality services, the government policy reward is *W*_1_, farmers do not speculate when joining integrated service organizations, and the policy reward is *W*_2_. If integrators provide inferior services, they will be punished as *P*_1_, and farmers' speculative behavior will be punished as *P*_2_. Regulatory costs arising from strict regulation are recorded as *C*_3_. When the government agriculture-related departments carry out loose supervision, there is no reward and punishment and no supervision cost.

**Hypothesis 6 .**

Integrators provide high-quality services, improve agricultural production efficiency, and improve the quality of agricultural products. For example, information services make agricultural products traceable and gain more trust from consumers, thus bringing social benefits to the government, which is recorded as *S*_*g*_. Integrators provide inferior services, join farmers to adopt speculative strategies, and join integrated organizations to become a mere formality, which affects the whole group of farmers' bad cognition of integrators. The resulting government governance cost is *M*_3_. If the government agriculture-related departments are still not strictly supervised at this time, they will be punished by their superior departments for their ineffective supervision, which will be recorded as *P*_3_ and *P*_3_ > *C*_3_.

### 2.3. Modeling

According to the above assumptions, this paper analyzes the corresponding benefits of integrators, farmers, and government agriculture-related departments under various strategy combinations, and gives a tripartite mixed strategy game matrix, which is shown in Table 1. When integrators choose to provide high-quality service strategy, farmers join the scale service system without speculation, and agriculture-related government departments carry out strict supervision; then, integrators' income is *R*_1_ − *C*_1*h*_+*W*_1_, farmers' income is *R*_2_+*R*_2*i*_+*W*_2_, and agriculture-related government departments' economic income is *S*_3_ − *C*_3_ − *W*_1_ − *W*_2_.

## 3. Model Analysis

### 3.1. Replication Dynamic Analysis

#### 3.1.1. Replication Dynamic Analysis of Integrators

The expected income of integrators providing high-quality services to farmers is *U*_11_, the expected income of providing poor-quality services to farmers is *U*_12_, and the average expected income is *U*_1_, which are, respectively, as follows:

(1) $$\begin{array}{c} U_{11}=yz\left(R_{1}-C_{1h}+W_{1}\right)+y\left(1-z\right)\left(R_{1}-C_{1h}\right)+z\left(1-y\right)\left(R_{1}-C_{1h}+W\right)+\left(1-y\right)\left(1-z\right)\left(R_{1}-C_{1h}\right)\text{,}\\ U_{12}=yz\left(-C_{1l}-C_{1s}-P_{1}\right)+y\left(1-z\right)\left(-C_{1l}-C_{1s}\right)+z\left(1-y\right)\left(R_{1}-C_{1l}-C_{1c}-C_{1s}-P_{1}\right)+\left(1-y\right)\left(1-z\right)\left(R_{1}-C_{1l}-C_{1c}-C_{1s}\right)\text{.}\\ U_{1}=xU_{11}+\left(1-x\right)U_{12}\text{.} \end{array}$$

The replication dynamic equation of integrator strategy selection is as follows: $\begin{array}{c} F\left(x\right)=dx/dt=x\left(U_{11}-U_{1}\right)=x\left(x-1\right)\left(U_{12}-U_{11}\right)\\ =x\left(x-1\right)\left[C_{1h}-C_{1l}-C_{1c}-C_{1s}-y\left(R_{1}-C_{1c}\right)-z\left(W_{1}+P_{1}\right)\right] \end{array}$

So, there are the following:

(2) $$\begin{array}{c} F\prime \left(x\right)=\frac{dF\left(x\right)}{dx}=\left(2x-1\right)\left[C_{1h}-C_{1l}-C_{1c}-C_{1s}-y\left(R_{1}-C_{1c}\right)-z\left(W_{1}+P_{1}\right)\right]\text{.} \end{array}$$

According to the stability theorem of differential equation, the probability of *F*′(*x*) < 0 integrator providing quality service is stable only if *F*(*x*)=0 is satisfied.

Let *Y*(*y*)=*C*_1*h*_ − *C*_1*l*_ − *C*_1*c*_ − *C*_1*s*_ − *y*(*R*_1_ − *C*_1*c*_) − *z*(*W*_1_+*P*_1_), then *∂Y*(*y*)/*∂y*=−(*R*_1_ − *C*_1*c*_) < 0, and we can see that *Y*(*y*) is a decreasing function.

Then, when *y*=*y*^*∗*^=[*C*_1*h*_ − *C*_1*l*_ − *C*_1*c*_ − *C*_1*s*_ − *z*(*W*_1_+*P*_1_)]/(*R*_1_ − *C*_1*c*_), any value of *x* has *F*(*x*)=0 and *F*′(*x*) ≡ 0, and the equation is stable, that is, any strategy of integrator is stable under this condition, and the probability of providing high-quality service will not change with time. When *y* ≠ *y*^*∗*^, *x*=0, or *x*=1, there are *F*(*x*)=0 and *F*′(*x*) symbols divided into the following two cases:

① When 0 < *y* < *y*^*∗*^, and *Y*(*y*) > 0, then *F*′(*x*)*|*_*x*=0_ < 0, *F*′(*x*)*|*_*x*=1_ < 0, and *x*=1 is the evolutionary stable point, that is, when the probability of farmers choosing not to speculate is less than *y*^*∗*^, the evolutionary stable strategy of integrators is to provide inferior services
② When *y*^*∗*^ < *y* < 1, and *Y*(*y*) < 0, then *F*′(*x*)*|*_*x*=0_ > 0, *F*′(*x*)*|*_*x*=1_ < 0, and *x*=1 is the evolutionary stable point, that is, when the probability of farmers choosing not to speculate is greater than *y*^*∗*^, the evolutionary stable strategy of integrators is to provide high-quality services

From the function *Y*(*y*), it can also be concluded that when 0 < *z* < [*C*_1*h*_ − *C*_1*l*_ − *C*_1*c*_ − *C*_1*s*_ − *y*(*R*_1_ − *C*_1*c*_)]/(*W*_1_+*P*_1_), 0 < *y* < *y*^*∗*^, and *x*=0 integrators provide inferior services, it is an evolutionary equilibrium strategy. When *y*^*∗*^ < *y* < 1, 1 > *z* > [*C*_1*h*_ − *C*_1*l*_ − *C*_1*c*_ − *C*_1*s*_ − *y*(*R*_1_ − *C*_1*c*_)]/(*W*_1_+*P*_1_), and *x*=1 integrators provide high-quality services, it is an evolutionary equilibrium strategy. That is to say, with the gradual increase in *y* and *z*, the evolution strategy of integrators has gradually evolved from *x*=0 (providing inferior services) to *x*=1 (providing superior services).  Corollary 1 can be obtained from this.

**Corollary 1 .**

In the evolution process, the probability of integrators providing high-quality services increases with the increase in the probability of farmers not speculating and the probability of strict supervision by government agriculture-related departments.

Corollary 1 shows that government departments want to improve the probability of integrators providing quality services by strengthening the supervision of government departments related to agriculture and also by reducing farmers' speculation. Government agriculture-related departments should strictly supervise when formulating various reward and punishment policies, and ensure that rewards really serve agricultural production, punish false speculation, and urge integrators to provide quality services to farmers. Government departments can ensure the accuracy and clarity of farmers' access to integrated production service information through publicity, informatization, and other measures, and eliminate farmers' uncertain intentions. Speculation will suffer losses, and it is in the best interests of farmers not to speculate.

The probability of integrators providing high-quality services is recorded as *K*_*i*1_, and the probability of providing inferior services is recorded as *K*_*i*2_, so there are the following:

(3) $$\begin{array}{c} K_{i2}=\overset{1}{\underset{0}{\int }}\overset{1}{\underset{0}{\int }}\frac{C_{1h}-C_{1l}-C_{1c}-C_{1s}-z\left(W_{1}+P_{1}\right)}{R_{1}-C_{1c}}dxdz=\frac{\left.2\left(C_{1h}-C_{1l}-C_{1c}-C_{1s}\right)-\left(W_{1}+P_{1}\right)\right)}{2\left(R_{1}-C_{1c}\right)}K_{i1}=1-K_{x2}=\frac{2\left(R_{1}-C_{1h}+C_{1l}+C_{1s}\right)+\left(W_{1}+P_{1}\right)}{2\left(R_{1}-C_{1c}\right)}\text{.} \end{array}$$

It can be concluded that

(4) $$\begin{array}{c} \frac{\partial K_{i1}}{\partial C_{1s}}>0,\frac{\partial K_{i1}}{\partial C_{1c}}>0,\frac{\partial K_{i1}}{\partial }\left(W_{1}+P_{1}\right)>0,\frac{\partial K_{i1}}{\partial }\left(C_{1h}-C_{1l}\right)<0_{。}\text{.} \end{array}$$

Because of 0 ≤ *K*_*i*1_ ≤ 1, *C*_1*h*_ − (*C*_1*l*_+*C*_1*s*_+*W*_1_+*P*_1_/2) ≥ *C*_1*c*_, and then, *∂K*_*i*1_/*∂R*_1_ > 0.  Corollary 2 can be drawn from the above analysis.

**Corollary 2 .**

The probability of providing high-quality services by integrators is directly proportional to the income of integrated services, lobbying costs, speculative costs, and government rewards and punishments, and inversely proportional to the difference between good and bad service costs.

It can be seen from Corollary 1 that if the service income of integrators can be guaranteed, it is beneficial to promote the high-quality service supply of integrators. The government can reduce the service cost of integrators, improve the service income of integrators, and promote the motivation of integrators to provide quality services for farmers through rural infrastructure construction and information construction. At the same time, the government can also promote integrators to provide high-quality agricultural production services by improving rewards and punishments.

#### 3.1.2. Dynamic Analysis of Replication of Farmers

The expected returns of nonspeculation and speculation of farmers are *U*_21_ and *U*_22_, respectively, and their average expected returns are *U*_2_, which are as follows:

(5) $$\begin{array}{c} U_{21}=xz\left(R_{2}+R_{2i}+W_{2}\right)+x\left(1-z\right)\left(R_{2}+R_{2i}\right)+z\left(1-x\right)\left(R_{2}-R_{2\;d}+W_{2}\right)\text{,}\\ U_{22}=xz\left(R_{2}+R_{2i}-C_{2}-P_{2}\right)+x\left(1-z\right)\left(R_{2}+R_{2i}-C_{2}\right)+\left(1-x\right)\left(1-z\right)\left(R_{2}-R_{2\;d}\right)+z\left(1-x\right)\left(R_{2}-R_{2\;d}-C_{2}+C_{1c}-P_{2}\right)+\left(1-x\right)\left(1-z\right)\left(R_{2}-R_{2\;d}+C_{1c}-C_{2}\right)\text{.}\\ U_{22}=xz\left(R_{2}+R_{2i}-C_{2}-P_{2}\right)+x\left(1-z\right)\left(R_{2}+R_{2i}-C_{2}\right)+\left(1-x\right)\left(1-z\right)\left(R_{2}-R_{2\;d}\right)+z\left(1-x\right)\left(R_{2}-R_{2\;d}-C_{2}+C_{1c}-P_{2}\right)+\left(1-x\right)\left(1-z\right)\left(R_{2}-R_{2\;d}+C_{1c}-C_{2}\right)\text{.} \end{array}$$

The replication dynamic equation of farmers' strategy choice is as follows:

*F*(*y*)=*dy*/*dt*=*y*(*U*_21_ − *U*_2_)=*y*(*y* − 1)(*U*_22_ − *U*_21_)=*y*(*y* − 1)[(*C*_1*c*_ − *C*_2_) − *xC*_1*c*_ − *z*(*W*_2_+*P*_2_)]. Then, it can be concluded that

(6) $$\begin{array}{c} F^{\prime }\left(y\right)=\frac{dF\left(y\right)}{dy}=\left(2y-1\right)\left[\left(C_{1c}-C_{2}\right)-xC_{1c}-z\left(W_{2}+P_{2}\right)\right]\text{.} \end{array}$$

According to the stability theorem of differential equation, the probability of farmers not speculating in *F*(*y*)=0 and *F*′(*y*) < 0 is stable only.

Let *Z*(*z*)=(*C*_1*c*_ − *C*_2_) − *xC*_1*c*_ − *z*(*W*_2_+*P*_2_), *∂Z*(*z*)/*∂z*=−(*W*_2_+*P*_2_) < 0, and *Z*(*z*) be a decreasing function.

Then, when *z*=*z*^*∗*^=[(*C*_1*c*_ − *C*_2_) − *xC*_1*c*_]/(*W*_2_+*P*_2_), any value of *y* has *F*(*y*)=0 and *F*′(*y*) ≡ 0, and the equations are stable, that is, in this case, any probability value of farmers is stable, and whether farmers speculate or not will not change with time. When *z* ≠ *z*^*∗*^, *y*=0, or *y*=1, the symbols of *F*(*y*)=0 and *F*′(*y*) are divided into the following two cases:

① When 0 < *z* < *z*^*∗*^, and *Z*(*z*) > 0, then *F*′(*y*)|_*y*=0_ < 0, *F*′(*y*)|_*y*=1_ > 0, and *y*=0 is the evolutionary stability point, that is, when the probability of strict supervision by agriculture-related government departments is less than *z*^*∗*^, the evolutionary stability strategy of farmers is to choose speculation
② When *z*^*∗*^ < *z* < 1, and *Z*(*z*) < 0, then *F*′(*y*)|_*y*=0_ < 0, *F*′(*y*)|_*y*=1_ < 0, and *y*=1 is the evolutionary stability point, that is, when the probability of strict supervision by agriculture-related government departments is greater than *z*^*∗*^, the evolutionary stability strategy of farmers is not speculative

From the function *Z*(*z*), it can be seen that when 0 < *x* < [(*C*_1*c*_ − *C*_2_) − *z*(*W*_2_+*P*_2_)]/*C*_1*c*_, 0 < *z* < *z*^*∗*^, and *y*=0 farmers choose speculation, it is an evolutionary stable strategy. When [(*C*_1*c*_ − *C*_2_) − *z*(*W*_2_+*P*_2_)]/*C*_1*c*_ < *x* < 1, *z*^*∗*^ < *z* < 1, and *y*=1 farmers choose not to speculate, it is an evolutionary stable strategy. That is, with the increase in *x* and *z*, the probability *y* of farmers choosing not to speculate increases.  Corollary 3 can be obtained from this.

**Corollary 3 .**

In the evolution process, the probability of farmers not speculating increases with the increase in the probability of integrators providing high-quality services and the probability of strict supervision by government agriculture-related departments.

From Corollary 3, it can be concluded that farmers' speculative behavior is related to the strategic choice of integrators and government agriculture-related departments. Government agriculture-related departments strengthen supervision, reward and punishment are well founded, integrators provide high-quality agricultural production services for farmers, and farmers can also refuse speculative behavior. Therefore, the scale operation of agricultural socialized service should run healthily and serve farmers' production. The agriculture-related departments of the government need to strengthen supervision and urge integrators to provide high-quality services, so as to gain farmers' recognition, avoid speculation, and form a good scale operation system of agricultural socialized service.

If the probability of farmers refusing speculation is recorded as *K*_*p*1_ and the probability of farmers speculating is recorded as *K*_*p*2_, there are the following:

(7) $$\begin{array}{c} K_{p2}=\overset{1}{\underset{0}{\int }}\overset{\left(C_{1c}-C_{2}/C_{1c}\right)}{\underset{0}{\int }}\frac{\left(C_{1c}-C_{2}\right)-xC_{1c}}{W_{2}+P_{2}}dxdy=\frac{{\left(C_{1c}-C_{2}\right)}^{2}}{2\left(W_{2}+P_{2}\right)C_{1c}}K_{p1}=1-K_{p2}=1-\frac{{\left(C_{1c}-C_{2}\right)}^{2}}{2\left(W_{2}+P_{2}\right)C_{1c}}\text{.} \end{array}$$

They are available as follows: *∂K*_*p*1_/*∂C*_2_=*C*_1*c*_ − *C*_2_/(*W*_2_+*P*_2_)*C*_1*c*_, *∂K*_*p*1_/*∂*(*W*_2_+*P*_2_)=*C*_1*c*_ − *C*_2_/2(*W*_2_+*P*_2_)^2^*C*_1*c*_, and *∂K*_*p*1_/*∂C*_1*c*_=*C*_2_^2^ − *C*_1*c*_^2^/2(*W*_2_+*P*_2_)*C*_1*c*_^2^ when *C*_1*c*_ > *C*_2_, *∂K*_*p*1_/*∂C*_2_ > 0, *∂K*_*p*1_/*∂*(*W*_2_+*P*_2_) > 0, and *∂K*_*p*1_/*∂C*_1*c*_ < 0, from which the following inference 4 can be obtained.

**Corollary 4 .**

When the lobbying cost of integrators is higher than the speculative cost of farmers, the probability of farmers choosing not to speculate increases with the increase in speculative cost and rewards and punishments of government agriculture-related departments, but decreases with the increase in lobbying cost of integrators.

Corollary 4 shows that whether farmers choose to speculate is not only related to their speculative costs, but also related to the lobbying costs of integrators and the rewards and punishments of government related to agriculture. The greater the cost of farmers' speculation, the smaller the possibility of farmers' speculation; the higher the lobbying cost of integrators, the greater the possibility of farmers' speculation; and the greater the rewards and punishments of government departments related to agriculture, the less likely it is for farmers to speculate. Therefore, in order to put an end to farmers' speculative behavior, governments at all levels can improve rewards and punishments through strict supervision, and can also reduce information flow costs, increase information transparency, and enhance credit management through rural informatization construction, thus reducing integrator lobbying costs and increasing farmers' speculative costs.

#### 3.1.3. Replication Dynamic Analysis of Government Agriculture-Related Departments

The expected income of government agriculture-related departments in choosing strict supervision and loose supervision strategies is *U*_31_ and *U*_32_, respectively, and their average expected income is *U*_3_, so there are the following:

(8) $$\begin{array}{c} U_{31}=xy\left(-C_{3}-W_{1}-W_{2}+S_{3}\right)+x\left(1-y\right)\left(-C_{3}-W_{1}+P_{2}+S_{3}\right)+y\left(1-x\right)\left(-C_{3}+P_{1}-W_{2}\right)+\left(1-x\right)\left(1-y\right)\left(-C_{3}+P_{1}+P_{2}-M_{3}\right)\text{.}\\ U_{32}=xyS_{3}+x\left(1-y\right)S_{3}+\left(1-x\right)\left(1-y\right)\left(-M_{3}-P_{3}\right)\text{,}\\ U_{3}=zU_{31}+\left(1-z\right)U_{32}\text{.} \end{array}$$

The replication dynamic equation of government agriculture-related departments is as follows:

(9) $$\begin{array}{c} F\left(z\right)=dz/dt=z\left(U_{31}-U_{3}\right)=z\left(z-1\right)\left(U_{32}-U_{31}\right)\\ =z\left(z-1\right)\left[C_{3}-P_{1}-P_{2}-P_{3}+x\left(W_{1}+P_{1}+P_{3}\right)+y\left(W_{2}+P_{2}+P_{3}\right)-xyP_{3}\right]\text{.} \end{array}$$

Then, it can be concluded that

(10) $$\begin{array}{c} F^{\prime }\left(z\right)=\frac{dF\left(z\right)}{dz}=\left(2z-1\right)\left[C_{3}-P_{1}-P_{2}-P_{3}+x\left(W_{1}+P_{1}+P_{3}\right)+y\left(W_{2}+P_{2}+P_{3}\right)-xyP_{3}\right]\text{.} \end{array}$$

According to the stability theorem of differential equation, only when *F*(*z*)=0 and *F*′(*z*) < 0, the probability of strict supervision by agriculture-related government departments is in a stable state.

Let *X*(*x*)=[*C*_3_ − *P*_1_ − *P*_2_ − *P*_3_+*x*(*W*_1_+*P*_1_+*P*_3_)+*y*(*W*_2_+*P*_2_+*P*_3_) − *xyP*_3_], and *∂X*(*x*)/*∂x*=(*W*_1_+*P*_1_+*P*_3_) − *yP*_3_ > 0, that is, *X*(*x*) monotone increases function with respect to *x*.

Then, when *x*=*x*^*∗*^=[*P*_1_+*P*_2_+*P*_3_ − *C*_3_ − *y*(*W*_2_+*P*_2_+*P*_3_)][(*W*_1_+*P*_1_+*P*_3_) − *yP*_3_], any value of *z* has *F*(*z*)=0 and *F*′(*z*) ≡ 0, and the equations are stable, that is, any probability value of strict supervision by agriculture-related government departments is stable, and the probability of strict supervision by agriculture-related government departments does not change with time. When *x* ≠ *x*^*∗*^, *z*=0, or *z*=1 all have *F*(*z*)=0, *F*′(*z*) symbols are divided into the following two cases:

① When 0 < *x* < *x*^*∗*^, *X*(*x*) < 0, *F*′(*z*)|_*z*=0_ > 0, and *F*′(*z*)|_*z*=1_ < 0, *z*=1 is the evolutionary stability point, that is, when the probability of integrators providing high-quality services is less than *x*^*∗*^, the evolutionary stability strategy of agriculture-related government departments is to choose strict supervision
② When *x*^*∗*^ < *x* < 1, and *X*(*x*) < 0, then *F*′(*z*)|_*z*=0_ < 0, *F*′(*z*)|_*z*=1_ > 0, and *z*=0 is the evolutionary stability point, that is, when the probability of integrators choosing to provide high-quality services is greater than *x*^*∗*^, the evolutionary stability strategy of agriculture-related government departments is loose supervision

From the function *X*(*x*), we can see that when 0 < *y* < [*P*_1_+*P*_2_+*P*_3_ − *C*_3_ − *x*(*W*_1_+*P*_1_+*P*_3_)]/(*W*_2_+*P*_2_+*P*_3_ − *xP*_3_), 0 < *x* < *x*^*∗*^, and *z*=1, government agriculture-related departments choose strict supervision that is an evolutionary stable strategy. When *x*^*∗*^ < *x* < 1, [*P*_1_+*P*_2_+*P*_3_ − *C*_3_ − *x*(*W*_1_+*P*_1_+*P*_3_)]/(*W*_2_+*P*_2_+*P*_3_ − *xP*_3_) < *y* < 1, and *z*=0 government agriculture-related departments choose loose supervision, it is their evolutionary stability strategy. That is, with the increase in *x* and *y*, the probability of strict government supervision decreases from *z*=1 to *z*=0, so *z* decreases with the increase in *x* and *y*. From this, we can get the following inference 5.

**Corollary 5 .**

In the evolution process, the probability of strict supervision by government agriculture-related departments decreases with the increase in the probability of integrators providing high-quality services and the probability of farmers not speculating.

Corollary 5 shows that the probability of strict supervision by government departments related to agriculture depends on the probability that integrators provide high-quality services and farmers do not speculate. When integrators provide quality services and farmers do not speculate, the government agriculture-related departments will not carry out strict supervision; when integrators provide inferior services and farmers' speculation is serious, the government agriculture-related departments will implement strict supervision. Therefore, the government agriculture-related departments, integrators, and farmers present a dynamic balance, and the decision-making of whether the government agriculture-related departments strictly supervise changes with the changes in integrators and farmers' behaviors, and the three parties present a dynamic balance.

If the probability of strict supervision by government agriculture-related departments is recorded as *K*_*g*1_ and the probability of loose supervision is recorded as *K*_*g*2_, then there are the following:

(11) $$\begin{array}{c} K_{g1}=\overset{1}{\underset{0}{\int }}\overset{1}{\underset{0}{\int }}\frac{P_{1}+P_{2}+P_{3}-C_{3}-y\left(W_{2}+P_{2}+P_{3}\right)}{\left(W_{1}+P_{1}+P_{3}\right)-yP_{3}}dydz=\frac{P_{1}+P_{2}+P_{3}}{P_{3}}-\left[\frac{W_{1}+W_{2}+C_{3}}{P_{3}}+\frac{\left(W_{2}+P_{2}\right)\left(W_{1}+P_{1}\right)}{P_{3}^{2}}\right]\ln\;\left(1+\frac{P_{3}}{W_{1}+P_{1}}\right)\text{.}\\ K_{g2}=\left[\frac{W_{1}+W_{2}+C_{3}}{P_{3}}+\frac{\left(W_{2}+P_{2}\right)\left(W_{1}+P_{1}\right)}{P_{3}^{2}}\right]\ln\;\left(1+\frac{P_{3}}{W_{1}+P_{1}}\right)-\frac{P_{1}+P_{2}}{P_{3}}\text{.} \end{array}$$

### 3.2. Stability Strategy Analysis of Tripartite Agent Evolutionary Game

According to the replication dynamic analysis of the above three parties, the local equilibrium points of agricultural socialized service scale management system can be obtained when *F*(*x*)=0, *F*(*y*)=0, and *F*(*z*)=0 are *E*_1_(0,0,0), *E*_2_(1,0,0), *E*_3_(0,1,0), *E*_4_(0,0,1), *E*_5_(1,1,0), *E*_6_(1,0,1), *E*_7_(0,1,1), and *E*_8_(1,1,1). The Jacobi matrix of the tripartite replication dynamical system is as follows:

(12) $$\begin{array}{c} J=\left[\begin{array}{ccc} \frac{\partial F\left(x\right)}{\partial x} & \frac{\partial F\left(x\right)}{\partial y} & \frac{\partial F\left(x\right)}{\partial z}\\ \frac{\partial F\left(y\right)}{\partial x} & \frac{\partial F\left(y\right)}{\partial y} & \frac{\partial F\left(y\right)}{\partial z}\\ \frac{\partial F\left(z\right)}{\partial x} & \frac{\partial F\left(z\right)}{\partial y} & \frac{\partial F\left(z\right)}{\partial z} \end{array}\right]\\ =\left[\begin{array}{ccc} \left(2x-1\right)\left[C_{1h}-C_{1l}-C_{1c}-C_{1s}-y\left(R_{1}-C_{1c}\right)-z\left(W_{1}+P_{1}\right)\right] & x\left(x-1\right)\left(C_{1c}-R_{1}\right) & x\left(1-x\right)\left(W_{1}+P_{1}\right)\\ y\left(1-y\right)C_{1c} & \left(2y-1\right)\left[\left(C_{1c}-C_{2}\right)-xC_{1c}-z\left(W_{2}+P_{2}\right)\right] & y\left(1-y\right)\left(W_{2}+P_{2}\right)\\ z\left(z-1\right)\left(W_{1}+P_{1}+P_{3}\right) & z\left(1-z\right)\left(W_{2}+P_{2}+P_{3}\right) & \left(2z-1\right)\left[C_{3}-P_{1}-P_{2}-P_{3}+x\left(W_{1}+P_{1}+P_{3}\right)+y\left(W_{2}+P_{2}+P_{3}\right)-xyP_{3}\right] \end{array}\right]\text{.} \end{array}$$

According to the Lyapunov indirect method, if the eigenvalues of Jacobi matrix *J* are all negative, the equilibrium point is evolutionary stability strategy (ESS). If at least one eigenvalue of the *J* matrix is positive, the equilibrium point is unstable. *J* Matrix has the eigenvalue whose real part is zero, and the other eigenvalues have the negative real part, and then, the equilibrium point is in the critical state, and the stability cannot be determined by the sign of the eigenvalue. The eigenvalues of the Jacobi matrix corresponding to each equilibrium point are shown in Table 2.

The symbols of eigenvalues of the Jacobi matrix at each equilibrium point are analyzed according to Table 2. According to Hypothesis 3, *C*_1*l*_ + *C*_1*c*_ + *C*_1*s*_ − *C*_1*h*_ < 0. Generally speaking, the speculative cost of farmers is less than the lobbying cost of integrators, that is, *C*_2_ − *C*_1*c*_ < 0, and the strict supervision cost of the government is less than the sum of the punishments of the three parties, that is, *C*_3_ − *P*_1_ − *P*_2_ − *P*_3_ < 0. The sign of *P*_2_ − *C*_3_ − *W*_1_ can be positive or negative and cannot be determined. Then, the eigenvalues of equilibrium point *E*(0,0,0) and *E*(1,0,0) Jacobi matrix are signed as “−, −, +” and “+, +, × (uncertain),” *E*(0,0,0) is the unstable point of the system, and *E*(1,0,0) is the unstable point of the system or saddle point. Obviously, *C*_1*l*_ + *C*_1*s*_ − *C*_1*h*_ + *R*_1_ > 0, −*C*_2_ + *C*_1*c*_ > 0, and *P*_1_ − *C*_3_ − *W*_2_ symbols are uncertain, so *E*_3_(0,1,0).

When *C*_1*l*_+*C*_1*c*_+*C*_1*s*_ − *C*_1*h*_+*W*_1_+*P*_1_ < 0 and*C*_2_ − *C*_1*c*_+*W*_2_+*P*_2_ < 0, the sign of the eigenvalue of *E*_4_(0,0,1) Jacobi matrix is “−, −, −,” and *E*_4_(0,0,1) is the evolutionary equilibrium point (ESS) of the system. *C*_1*h*_ − *C*_1*l*_ − *C*_1*s*_ − *R*_1_ < 0, and obviously *E*_5_(1,1,0) is the evolutionary equilibrium point (ESS) of the system. Because the sign of *C*_3_+*W*_1_ − *P*_2_ and *C*_3_+*W*_2_ − *P*_1_ cannot be determined, the sign of eigenvalue of *E*_6_(1,0,1) and *E*_7_(0,1,1) Jacobi matrix is “+, +, ×” and “+, +, ×,” respectively, then *E*_6_(1,0,1) and *E*_7_(0,1,1) are unstable points or saddle points of the system. Obviously, the sign of the eigenvalue of *E*_8_(1,1,1) Jacobi matrix is “+, +, −,” which is the unstable point of the system. The real part symbol and stability arrangement of eigenvalues of each equilibrium point are shown in Table 3.

According to the analysis in Table 2, it can be concluded that *E*_5_(1,1,0) is the evolutionary stable point (ESS). When *C*_1*l*_+*C*_1*c*_+*C*_1*s*_ − *C*_1*h*_+*W*_1_+*P*_1_ < 0 and *C*_2_ − *C*_1*c*_+*W*_2_+*P*_2_ < 0, *E*_4_(0,0,1) is also the evolutionary stable point (ESS).  Corollary 6 can be obtained from this.

**Corollary 6 .**

*E*_5_(1,1,0) is the evolutionary stable point of the replicated dynamic system. When *C*_1*l*_+*C*_1*c*_+*C*_1*s*_ − *C*_1*h*_+*W*_1_+*P*_1_ < 0 and *C*_2_ − *C*_1*c*_+*W*_2_+*P*_2_ < 0, *E*_4_(0,0,1) is also the stable point of replicating the dynamic system.

Corollary 6 shows that (high-quality service, nonspeculation, and loose supervision) must be a stable strategic combination of the dynamic system of supply and demand of agricultural socialized services composed of integrators, farmers, and agriculture-related government departments. However, when the cost of providing high-quality service is too high (greater than the sum of low-quality service cost, lobbying cost, speculative cost, and government rewards and punishments) and lobbying cost is larger (greater than the sum of farmers' speculative cost and government rewards and punishments), (inferior service, speculation, and strict supervision) will also be the stable strategy combination of the system. Obviously, the combination of strategies (quality service, nonspeculation, and loose supervision) is superior to the combination of strategies (poor service, speculation, and strict supervision). Therefore, the agriculture-related government departments crack down on speculative activities, increase speculative costs, improve rewards and punishments, and promote the evolution of the agricultural service scale management system to the strategy combination of (high-quality service, nonspeculation, and loose supervision), thus providing strong support for the healthy development of agricultural production. However, the agricultural socialization service system is a complex system, and the influence of various factors on the main body of the system and the internal influence mechanism needs to be further studied.

## 4. Simulation Analysis

Combined with the parameter comparison among integrators, farmers, and agriculture-related government departments in reality, the value is assigned, and MATLAB2018 software is used for simulation demonstration to verify the effectiveness of the model. Under normal circumstances, the cost of providing high-quality services by integrators meets *C*_1*h*_ < *C*_1*l*_+*C*_1*c*_+*C*_1*s*_+*W*_1_+*P*_1_ (*∗*), and the lobbying cost meets *C*_1*c*_ < *C*_2_+*W*_2_+*P*_2_ (*∗∗*). Therefore, the parameters of the three participants are assigned as shown in Table 4, and the influence of the changes in each parameter on the evolution process and results is discussed, respectively.

### 4.1. Evolution Simulation of Tripartite Important Parameters

#### 4.1.1. Changes in Integrator Revenue

The integrator's income is the main influencing factor of its behavior. We analyze the influence of its change on the process and results of the evolutionary game, take *R*_1_ = 80, *R*_1_ = 100, and *R*_1_ = 120, respectively, and copy the simulation results of dynamic equations evolving with time as shown in Figure 2. It can be seen that with the increase of R1, the speed of system evolution to the stable point is accelerated; with the increasing probability of integrators providing quality services, the probability of strict supervision by agriculture-related government departments decreases. Therefore, in the early stage of service scale operation, when the service capacity of integrators is uneven and the probability of providing high-quality services is low, the government should strengthen supervision to ensure the benign operation of the agricultural production service system.

#### 4.1.2. Changes in the Cost of Providing Quality Services by Integrators

When integrators provide high-quality services and their costs are *C*_1*h*_=50, *C*_1*h*_=55, *C*_1*h*_=60, the simulation results of copying dynamic equations evolving with time are shown in Figure 3. In the process of system evolution to a stable point, with the reduction in service cost, the evolution speed of integrators providing high-quality services can be accelerated, the probability of integrators providing high-quality services increases, and the probability of strict government supervision decreases. Therefore, agriculture-related government departments can reduce the operating cost of integrators' scale services and promote the probability of integrators providing quality services by constructing service platforms and strengthening digital construction.

#### 4.1.3. Integrators' Lobby Cost Changes

When the lobbying cost of integrators is *C*_1*c*_ = 10, *C*_1*c*_ = 15, *C*_1*c*_ = 20, the simulation results of copying dynamic equations evolving with time are shown in Figure 4. It can be seen that the lobbying cost of integrators increases. When the probability of farmers not speculating and integrators providing high-quality services is low, the probability of strict government supervision rapidly rises. Until the probability of farmers not speculating and integrators providing high-quality services is high, the government gradually relaxes supervision and the probability of strict supervision drops to 0. Therefore, in the initial stage of agricultural scale service, integrators convince farmers in order to obtain preferential policies from the state; farmers are tempted by certain interests to speculate [20]. At this time, the agriculture-related government departments should strengthen supervision, so as to avoid collusion between integrators and farmers to obtain preferential policies from the state and damage the real agricultural production.

#### 4.1.4. Changes in Rewards and Punishments of Integrators

The government takes different rewards and penalties for integrators, *W*_1_=5, *W*_1_=15, *W*_1_=25 for rewards and *P*_1_=10, *P*_1_=20, *P*_1_=30 for penalties, and the evolutionary simulation results of their replication dynamic equations are shown in Figures 5 and 6. From the evolutionary simulation diagram, it can be seen that the characteristics of punishment and reward are similar: the punishment is increased, the scale service system evolves to a stable point faster, and the probability of government supervision is reduced. With the increase in incentives, the system also evolves to a stable point faster, and the probability of government supervision decreases. Reward is faster than punishment, which reduces the probability of strict government supervision to 0.

#### 4.1.5. Change in Farmers' Policy Incentives

The speculative cost of farmers takes different values *W*_2_=5, *W*_2_=10, *W*_2_=15, and the simulation results of copying the dynamic equation evolving with time are shown in Figure 7. In the process of system evolution to the stable point, the higher the farmer policy reward, the faster the system evolution to the stable point (1, 1, 0), and the smaller the probability of strict government supervision. Therefore, it can improve the reward level of farmers and promote the system to provide high-quality services to integrators; farmers do not speculate; and the government can relax supervision.

#### 4.1.6. Changes in Punishment by Higher-Level Governments

The supervision and punishment of higher-level government departments on agriculture-related government departments have a significant impact on the evolution of the scale service system. The higher-level government punishes different values *P*_3_=20, *P*_3_=30, *P*_3_=40 and copies the dynamic equation evolution simulation results as shown in Figure 8. The punishment of higher-level government increases, and the probability of strict supervision of agriculture-related government departments increases; with integrators providing high-quality services, the probability of farmers not speculating increases, while the probability of strict supervision by agriculture-related government departments decreases. Therefore, strengthening the supervision of higher-level government on the supervision of agriculture-related government departments is also conducive to the benign operation of the agricultural scale service system.

### 4.2. System Evolution Simulation under Different Conditions

The previous section analyzed the evolution of the system satisfying the (*∗*) and (*∗*) conditions, and this section discussed the evolution simulation of the agricultural scale service system satisfying the above two conditions and not satisfying the above two conditions. Table 4 shows the parameter assignments that meet the above conditions, and Table 5 shows the parameter assignments that do not meet the above two conditions.

The two sets of assignments evolved 50 times with time from different initial strategy combinations, and the simulation results are shown in Figures 9 and 10. It can be seen from the simulation results that when the conditions (*∗*) and (*∗*) are satisfied, that is, *C*_1*h*_ < *C*_1*l*_+*C*_1*c*_+*C*_1*s*_+*W*_1_+*P*_1_ and *C*_1*c*_ < *C*_2_+*W*_2_+*P*_2_ are satisfied, the system has only one evolutionary stable point (1, 1, 0), while when the above two conditions are not satisfied, the system has two evolutionary stable points (0, 0, 1) and (1, 1, 0). In other words, when the cost of providing high-quality services by integrators is small and lobbying is not of great benefit to farmers, the final evolution result of the scale service management system is (providing high-quality services, not speculating, and loose supervision). When the cost of providing high-quality services by integrators is too high, and lobbying farmers get enough benefits for farmers, the final evolution result of the scale service management system may be (providing inferior services, speculation, and strict supervision) or (providing high-quality services, no speculation, and loose supervision). Obviously, from the perspective of overall social benefits, the balanced result (providing high-quality services, not speculating, and loosening supervision) is better than (providing poor-quality services, speculating, and strictly supervising).

Many cases in agricultural practice have proved that when local governments combine capital and power in the countryside for performance [20] and take national preferential policies, or national preferential policies are captured by elites and are not implemented in common agricultural production activities, the healthy operation of scale services is seriously affected [22], and finally, a low-level balance (providing inferior services, speculation, and strict supervision) is formed, which damages the normal operating environment of agricultural production. Then, how to improve and promote the Pareto high-efficiency equilibrium (providing high-quality services, not speculating, and loosening supervision)? Zhang Weiying [31] pointed out that stable policies help people screen a specific Nash equilibrium among multiple equilibria by coordinating people's expectations. Therefore, what kind of policies should the government provide to guide the system to transform into Pareto high-efficiency equilibrium is a topic worthy of in-depth study in the follow-up.

## 5. Conclusions

This paper studies the evolutionary game of agricultural service scale management system composed of integrators, farmers, and agriculture-related government departments. By constructing the evolutionary game model of three parties, the stability and evolutionary results of the system under various strategies are analyzed, and the effectiveness of the evolutionary results is verified by simulation analysis. The main conclusions of this study include the following:

1. The dynamic changes in integrators, farmers, and agriculture-related government departments influence each other: the higher the probability that farmers do not speculate and agriculture-related government departments strictly supervise, the more integrators tend to provide high-quality services. The more integrators tend to provide quality services, the stricter the supervision of agriculture-related government departments, and the greater the probability of farmers not speculating. The higher the probability that farmers do not speculate and integrators provide high-quality services, the more the agriculture-related government departments tend to loosen supervision.
2. The probability of providing high-quality services increases with the increase in their own income, lobbying cost, speculative cost, and government rewards and punishments, and decreases with the increase in the cost difference between providing high-quality services and poor-quality services. The probability of nonspeculation of farmers is influenced by the government and integrators besides their own factors, which increases with the increase in their own speculative costs and rewards and punishments of agriculture-related government departments, and decreases with the increase in lobbying costs of integrators.
3. When the cost difference between high-quality service and low-quality service provided by integrators is small, there is only one tripartite scale service system evolution equilibrium among integrators, farmers, and agriculture-related government departments (providing high-quality service, not speculating, and loosening supervision). When there is a big cost difference between high-quality service and low-quality service (low-quality service, speculation, and strict supervision), it is also the evolutionary equilibrium of this system. The government should provide effective policies to guide the evolution of the system to a high-level stable state.

This study also has some limitations. First of all, the agricultural scale service system also includes upstream material suppliers, such as seeds and fertilizers, and downstream sellers, such as farmers' markets and supermarkets, which are not included in this system. Second, the results of system evolution are not only influenced by each other but also by external risks, which need further consideration. Finally, when the cost of the integrator to provide high-quality service is high, there is obvious Pareto improvement space for the two evolutionary equilibrium results. Social trust, long-term relationship, repeated game, and cooperation between parties may be the basis for guiding the system to evolve to high-level equilibrium, which still needs further research.

## Figures and Tables

**Figure 1:** Logical relationship of tripartite evolution of agricultural service scale operation.

**Figure 2:** Changes in integrator revenue.

**Figure 3:** Changes in the cost of providing quality services by integrators.

**Figure 4:** Changes in lobbying costs of integrators.

**Figure 5:** Changes in government incentives for integrators.

**Figure 6:** Changes in government penalties for integrators.

**Figure 7:** Changes in farmers' policy incentives.

**Figure 8:** Changes in punishment by higher-level governments.

**Figure 9:** Evolution results satisfying (*∗*) and (*∗∗*) conditions.

**Figure 10:** Evolution results that do not satisfy (*∗*) and (*∗∗*) conditions.

**Table 1:** Establishment of the payment matrix of the game model among integrators, farmers, and government departments related to agriculture.

Strategy combination	Integrator revenue	Farmer income	Income of agriculture-related government departments
High quality, not speculative, and strict	*R*_1_ − *C*_1*h*_+*W*_1_	*R*_2_+*R*_2*i*_+*W*_2_	−*C*_3_ − *W*_1_ − *W*_2_+*S*_3_
High quality, not speculative, and not strict	*R*_1_ − *C*_1*h*_	*R*_2_+*R*_2*i*_	*S*_3_
High quality, speculative, and strict	*R*_1_ − *C*_1*h*_+*W*_1_	*R*_2_+*R*_2*i*_ − *C*_2_ − *P*_2_	−*C*_3_ − *W*_1_+*P*_2_+*S*_3_
High quality, speculative, and not strict	*R*_1_ − *C*_1*h*_	*R*_2_+*R*_2*i*_ − *C*_2_	*S*_3_
Inferior, not speculative, and strict	−*C*_1*l*_ − *C*_1*s*_ − *P*_1_	*R*_2_ − *R*_2 *d*_+*W*_2_	−*C*_3_+*P*_1_ − *W*_2_
Inferior, not speculative, and not strict	−*C*_1*l*_ − *C*_1*s*_	*R*_2_ − *R*_2 *d*_	0
Inferior, speculative, and strict	*R*_1_ − *C*_1*l*_ − *C*_1*c*_ − *C*_1*s*_ − *P*_1_	*R*_2_ − *R*_2 *d*_ − *C*_2_+*C*_1*c*_ − *P*_2_	−*C*_3_+*P*_1_+*P*_2_ − *M*_3_
Inferior, speculative, and lax	*R*_1_ − *C*_1*l*_ − *C*_1*c*_ − *C*_1*s*_	*R*_2_ − *R*_2 *d*_+*C*_1*c*_ − *C*_2_	−*M*_3_ − *P*_3_

**Table 2:** Eigenvalues of the Jacobi matrix at each equilibrium point.

Equilibrium point	Eigenvalue *λ*_1_	Eigenvalue *λ*_2_	Eigenvalue *λ*_3_
*E*_1_(0,0,0)	*C*_1*l*_+*C*_1*c*_+*C*_1*s*_ − *C*_1*h*_	*C*_2_ − *C*_1*c*_	*P*_1_+*P*_2_+*P*_3_ − *C*_3_
*E*_2_(1,0,0)	*C*_1*h*_ − *C*_1*l*_ − *C*_1*c*_ − *C*_1*s*_	*C*_2_	*P*_2_ − *C*_3_ − *W*_1_
*E*_3_(0,1,0)	*C*_1*l*_+*C*_1*s*_ − *C*_1*h*_+*R*_1_	−*C*_2_+*C*_1*c*_	*P*_1_ − *C*_3_ − *W*_2_
*E*_4_(0,0,1)	*C*_1*l*_+*C*_1*c*_+*C*_1*s*_ − *C*_1*h*_+*W*_1_+*P*_1_	*C*_2_ − *C*_1*c*_+*W*_2_+*P*_2_	*C*_3_ − *P*_1_ − *P*_2_ − *P*_3_
*E*_5_(1,1,0)	*C*_1*h*_ − *C*_1*l*_ − *C*_1*s*_ − *R*_1_	−*C*_2_	−*C*_3_ − *W*_1_ − *W*_2_
*E*_6_(1,0,1)	*C*_1*h*_ − *C*_1*l*_ − *C*_1*c*_ − *C*_1*s*_ − *W*_1_ − *P*_1_	*C*_2_+*W*_2_+*P*_2_	*C*_3_+*W*_1_ − *P*_2_
*E*_7_(0,1,1)	*C*_1*l*_+*C*_1*s*_ − *C*_1*h*_+*W*_1_+*P*_1_+*R*_1_	*C*_1*c*_ − *C*_2_ − *W*_2_ − *P*_2_	*C*_3_+*W*_2_ − *P*_1_
*E*_8_(1,1,1)	*C*_1*h*_ − *C*_1*l*_ − *C*_1*s*_ − *W*_1_ − *P*_1_ − *R*_1_	−*C*_2_ − *W*_2_ − *P*_2_	*C*_3_+*W*_1_+*W*_2_

**Table 3:** Real part coincidence and stability of eigenvalues of equilibrium points.

Equilibrium point	Real part symbol	Stability conclusion
*E*_1_(0,0,0)	(−, −, +)	Unstable point
*E*_2_(1,0,0)	(+, +, ×)	Unstable point or saddle point
*E*_3_(0,1,0)	(+, +, ×)	Unstable point
*E*_4_(0,0,1)	(−, −, −)	ESS
*E*_5_(1,1,0)	(−, −, −)	ESS
*E*_6_(1,0,1)	(×, −, ×)	Unstable point
*E*_7_(0,1,1)	(+, ×, ×)	Unstable point
*E*_8_(1,1,1)	(−, −, +)	Unstable point

**Table 4:** Parameter assignment under (*∗*) and (*∗*) conditions.

Parameter	*R*_1_	*C*_1*h*_	*C*_1*l*_	*C*_1*c*_	*C*_1*s*_	*C*_2_	*W*_1_	*W*_2_	*P*_1_	*P*_2_	*C*_3_	*P*_3_
Assignment	80	60	5	20	5	5	15	10	20	10	10	30

**Table 5:** Parameter assignments that do not satisfy (*∗*) and (*∗∗*).

Parameter	*R*_1_	*C*_1*h*_	*C*_1*l*_	*C*_1*c*_	*C*_1*s*_	*C*_2_	*W*_1_	*W*_2_	*P*_1_	*P*_2_	*C*_3_	*P*_3_
Assignment	100	85	5	30	5	5	15	5	15	5	10	30

## Data Availability

The experimental data used to support the findings of this study are available from the corresponding author upon request.
